RETRACTED

# Effect of Cross Theoretical Model of Behaviour Change and Motivation Interview on Self-Management Behaviour

**DOI:** 10.1155/2022/3551167

**Published:** 2022-08-22

**Authors:** Hongxia Wang, Dongmei Li, Ye Xiong, Huijun Huang, Qiongshuang Hu, Weimei Zhang

**Affiliations:** ^1^Department of Nursing, The First Hospital Affiliated to Wenzhou Medical University, Ouhai District, Wenzhou 325000, Zhejiang Province, China; ^2^Department of Neurosurgery, The First Hospital of Wenzhou Medical University, Ouhai District, Wenzhou 325000, Zhejiang Province, China; ^3^Interventional Surgery Centre, The First Hospital of Wenzhou Medical University, Ouhai District, Wenzhou 325000, Zhejiang Province, China

## Abstract

**Objective:**

To evaluate the effects of a trans-theoretical model (TTM) of behavioural change plus motivational interviewing on self-management behavior and quality of life (QoL) in patients with intracranial aneurysm.

**Methods:**

A total of 94 patients with intracranial aneurysm treated in the First Affiliated Hospital of Wenzhou Medical University from 2019 to 04/2021-04 were retrospectively analyzed. Among them, 49 patients used TTM + motivational interview as the observation group (Obs group), and 45 patients used the traditional method as the control group (Con group). The Self-Management Behavior Scale for Patients with Intracranial Aneurysm was used for analyzing the changes in the self-management behavior of the two groups of patients, and the MOS 36-item Short Form Health Survey (SF-36) was used to analyze the changes in the QoL of the patients. The incidence of adverse events after 6 months of intervention was counted. In addition, the Barthel Index (BI) and Montreal Cognitive Assessment Scale (MOCA) were used to evaluate the recovery effects of patients. Logistic regression was conducted for analyzing the risk factors of adverse cerebrovascular events.

**Results:**

After treatment, the Con group got lower self-management behavior score than the Obs group (*P* < 0.05), and also got lower SF-36 scores, BI, and MOCA scores than the Obs group (*P* < 0.05). Age and a history of hypertension were independent risk factors for adverse events. The Hosmer–Lemeshow test was adopted for testing the goodness of fit of the regression equation (*P*=0.903). With the established model, the area under the receiver operating characteristic curve for predicting adverse events in patients with intracranial aneurysm was determined to be 0.851, indicating that the model performed well as a risk prediction model.

**Conclusion:**

TTM + motivational interviewing can help improve the self-management behavior and QoL of patients with intracranial aneurysm without increasing the occurrence of adverse events.

RETRACTED

## 1. Introduction

Subarachnoid hemorrhage (SAH) is one frequently-seen acute cerebrovascular disease in clinical scenarios, with an incidence of 5–20/100,000, occupying 20% of hemorrhagic strokes, and over half of the survivors are accompanied by irreversible brain damage, suffering a terribly high disability rate and mortality rate [1]. Intracranial aneurysm is the primary cause of SAH [2]. Despite the consistent updating of the medical level, SAH still shows mortality as high as 20%. About one-third of the survivors suffer from chronic neurological deficits with cognitive dysfunction and thus require care from others. In addition, the population suffering from SAH tends to be younger, which brings a huge economic burden to families and society, and thus captures increasing attention from the medical community and the government [3]. Therefore, clinically, there exists an urgent need for a recovery plan to improve the condition of patients with it and enhance their self-care ability.

The trans-theoretical model (TTM) of behaviour change was put forward by Prochaska in 1982. It is a clinical method of healthy behaviour change and has been deemed as one of the most crucial theoretical health promotion models in the past 10 years [4]. Motivational interviewing was originally proposed by Miller, an American scholar, in 1983 as a simple intervention method for drinking problems and then developed and improved by Miller and Rollnick, a professor of clinical psychology in Britain [5]. Motivational interviewing is a patient-centered interpersonal communication method that changes patients' bad behaviours and solves their ambivalence by stimulating the intrinsic motivation of their behaviour changes [6]. Bassilios et al. [7] found through research on 49 patients sampled from three community psychiatric centers in Melbourne (Australia) that TTM can also help improve the patients' exercise level despite their high level of mental symptoms. According to another study, TTM lowered the risk of cardiovascular diseases by changing unhealthy behaviours and promoting the cultivation of healthy lifestyles [8]. However, the effects of TTM + motivational interviewing on the quality of life (QoL) and self-management behaviour of patients with intracranial aneurysm have yet to be studied.

Accordingly, this study applied TTM + motivational interviewing to patients with intracranial aneurysm to improve their self-management ability, relieve their stress reaction, improve their QoL, and promote their early return to society.

## 2. Methods and Data

### 2.1. Clinical Data

A total of 94 patients with intracranial aneurysm treated in The First Hospital Affiliated to Wenzhou Medical University between April 2019 and April 2021 were retrospectively analyzed. Among them, 49 patients were interviewed by TTM + motivational interviewing as an observation group (Obs group), and 45 patients by the traditional method as a control group (Con group). This study was conducted with the permission from the Medical Ethics Committee of the first affiliated Hospital of Wenzhou Medical University.

RETRACTED

### 2.2. Inclusion and Exclusion Criteria

#### 2.2.1. The Inclusion Criteria

Patients who met the American Heart Association/American Stroke Association guidelines [9]. Patients who were confirmed with a single intracranial aneurysm by computed tomography angiogram (CTA) or digital subtract angiography (DSA) and treated in our department. Patients who are able to cooperate with us to complete the investigation with clear conscious and normal verbal communication ability; patients ≥18 years old or ≤60 years old; and patients who signed informed consent forms after being apprised of the study.

#### 2.2.2. The Exclusion Criteria

Patients with malignant tumors or tumor metastases, patients with comorbid heart failure or other organic diseases, patients who dropped out of the study or who were unable to complete treatment during the study, patients with serious infections, and pregnant women.

### 2.3. Intervention Plan

#### 2.3.1. The Con group

Each patient was given routine health education for intracranial aneurysm according to the characteristics of his/her disease and condition, and encouraged to learn related posters (posters related to healthy diet and exercise management in ward corridors) and manuals. In addition, the patient was informed of the benefits of behaviour change so that the patient would voluntarily change bad behaviours or maintain healthy behaviours.

#### 2.3.2. The Obs group

Each patient was intervened by TTM + motivational interviewing additionally based on intervention to the Con group: (1) set up a TTM + motivational interviewing group and design a self-management behaviour scale for patients with intracranial aneurysm; (2) implement targeted intervention for patients by motivational interviewing-based health education after evaluating the behaviour stage of patients with the TTM-based phased change assessment questionnaire based on intervention to the Con group (Table 1).

### 2.4. Outcome Measures

Primary outcome measures: the self-management behavior scale of patients with intracranial aneurysm was used to analyze the changes of self-management behavior before treatment and after 3 months of treatment in the two groups, and the MOS36 short-term health survey (SF-36) was used for analyzing the changes in patients' QoL [10]. It is divided into six dimensions, with the highest score of 100 points. The higher the score, the more normal QoL. Adverse event rates were calculated 6 months after the intervention.

RETRACTED

Secondary outcome measures: the clinical data were also compared between the two groups. Additionally, Barthel index (BI) and Montreal cognitive assessment (MOCA) scale were used for evaluating the rehabilitation of patients [11, 12]. The total score of the BI score is 100, with a higher score indicating better ability of independent living activities. The total score of the MoCA score is 30, and a higher score indicates cognitive function and normal. Logistic regression was carried out to analyze the risk factors of adverse cerebrovascular events, and a regression model was established.

### 2.5. Statistical Analyses

This study adopted SPSS 20.0 (IBM Corp., Armonk, NY, USA) for data processing and graphpad prism 8 software data for visualization of data. Intergroup comparisons were performed via the independent sample *t* test, and intro-group comparisons were performed using the paired *t* test. Count data were analyzed by *χ*^2^ test. Logistic regression was used to analyze the risk factors of adverse cerebrovascular events. The Hosmer–Lemeshow test was adopted for testing the goodness of fit of the regression equation. The efficacy of adverse cerebrovascular events was analyzed by ROC curve. A *P*< value of 0.05 suggests a notable difference.

## 3. Results

### 3.1. Comparison of Clinical Data

Comparison of clinical data between the two groups revealed no notable difference between them in age, gender, body mass index (BMI), past medical history, and location of aneurysm (all *P* > 0.05, Table 2).

### 3.2. Changes of Self-Management Behaviours

According to a comparison of the results obtained by the self-management behaviour between the two groups prior and post-therapy, before treatment, the two groups were not greatly different regarding self-management behaviour scores (*P* > 0.05), while after treatment, the scores of the two groups were notably improved, with notably lower self-management behaviour scale scores in the Con group than those in the Obs group (*P* < 0.05, Figure 1).

### 3.3. Changes of QoL

According to the comparison of SF-36 scores prior- and post-therapy between the two groups, before therapy, the two groups were similar in SF-36 scores (*P* > 0.05); after therapy, the SF-36 scores of the two groups notably improved, with notably lower SF-36 scores in the Con group than those in the Obs group (*P* < 0.05, Figure 2).

### 3.4. Comparison of Rehabilitation

According to the comparison of BI and MOCA scores between the two groups prior- and post-therapy, before therapy, the two groups were similar in both BI and MOCA scores (*P* > 0.05); after therapy, both BI and MOCA scores of the two groups were notably improved, with notably lower BI and MOCA scores in the Con group than those in the Obs group (*P* < 0.05, Table 3, Figure 3).

RETRACTED

### 3.5. Incidence of Adverse Events

The comparison between the two groups in incidence of adverse events revealed no notable difference in the total incidence of adverse events between the Con group and Obs group (*P* > 0.05, Table 4).

### 3.6. Analysis of Risk Factors of Adverse Events

For understanding the risk factors of adverse events, patients were assigned to the occurrence group (*n* = 16) or the nonoccurrence group (*n* = 78) according to the adverse events. The clinical data of patients were collected and assigned and then subjected to logistic regression (*P* > 0.05, Table 5). All indexes were selected, and the entry method was used for analysis. According to the results, age, sex, and history of hypertension were the risk factors of adverse events. Then the backward LR was adopted for multivariate analysis, and the age and history of hypertension were discovered to be independent risk factors for adverse events (*P* > 0.05, Table 6). For further determining the value of age and history of hypertension in the occurrence of adverse events, a risk prediction equation was established: Logit *P* = −5.056 + 2.760 × *X*1 + 2.785 × *X*2. The Hosmer–Lemeshow test was adopted for testing the goodness of fit of the regression equation (*P*=0.903). With the established model, it was determined that the area under the ROC curve (AUC) for predicting adverse events in patients with intracranial aneurysm was 0.851 (Figure 2, Table 7, 95% CI: 0.7509–0.9519, *P* < 0.001), indicating the good performance of the model as a risk prediction model.

## 4. Discussion

Intracranial aneurysm is the local pathological expansion of intracranial blood vessels with a high mortality and disability rate, which can trigger cerebral hemorrhage in patients. For patients with intracranial aneurysm who suffer hemorrhage, the risk of rebleeding is high, which could bring serious adverse consequences [13]. According to studies, the recurrence rate of intracranial aneurysm after endovascular interventional therapy is up to 20.8%–36%, and patients who have risk factors including smoking, alcoholism, hypertension, diabetes mellitus, and hyperlipidemia often face risks of multiple or postoperative recurrence [14, 15]. The related factors of intracranial aneurysm rupture are not only bound up with the size and location of the intracranial aneurysm but also strongly bound up with patients' self-protection, emotional management, blood pressure control, medication compliance, and changes of bad living habits [16, 17].

RETRACTED

The aim of TTM is to provide targeted behavioural support according to the individual needs of the behaviour change object and to carry out health education in stages according to the patient's intention to change behaviours [18]. Motivational interviewing aims to help patients discover and overcome their contradictory psychological state based on effective communication so that they can better participate in the analysis and evaluation of intervention programs, better understand the risks and benefits of intracranial aneurysm, and thus benefit from behavioural changes [19, 20]. However, the effects of TTM + motivational interviewing in the management of intracranial aneurysm patients are still under investigation. Our study analyzed the effects of TTM + motivational interviewing on self-management behaviour and QoL of patients with intracranial aneurysm. According to the results, the self-behaviour management of patients in the Obs group was significantly improved after the application of TTM + motivational interviewing, which was higher than that of the Con group. Moreover, after therapy, the Obs group got a higher SF-36 score than the Con group, suggesting the function of TTM + motivational interviewing in effectively improving the self-management ability and QoL of patients with intracranial aneurysm. The primary reason may be as follows: with TTM + motivational interviewing, targeted behaviour change programs can be adopted at different stages according to the behaviour characteristics of patients at different stages to meet the needs of patients. In the preintention and intentional stages, the interviewees can guide the patients' self-management motivation by chatting, thus effectively improving the patients' self-management ability and QoL. Ream et al. [21] found that motivational interviewing by telephone can reduce the fatigue intensity, self-efficacy for fatigue, and anxiety level of patients with cancer. In addition, according to prior research, TTM + motivational interviewing can deliver favourable effects in preventing female osteoporosis [22], substance dependence such as ethanol drugs [23], human immunodeficiency virus infection [24], and cancer pain management. Our study has also verified the promotional role of TTM + motivational interviewing in improving the self-management behaviour and QoL of patients with intracranial aneurysm.

Moreover, the changes of rehabilitation in the two groups were compared prior- and post-treatment in our study. The Obs group got notably higher BI and MOCA scores than the Con group, indicating that TTM + motivational interviewing can also promote the postoperative rehabilitation of patients. The reasons are as follows: TTM + motivational interviewing is patient-centered, which aims to cultivate the disease management ability of patients and their nurses and promotes the change of patients' behaviour intention stage through health education by medical staff, thus improving the patients' behaviour, prognosis, and recovery. In addition, no notable difference was found in the incidence of adverse events between the two groups according to the 6-monthfollow-up in our study, indicating that TTM + motivational interviewing would not increase the incidence of adverse events in patients.

RETRACTED

Finally, the risk factors of patients' adverse events were analyzed. Through the established regression model, age and history of hypertension were discovered to be independent risk factors for adverse events in patients with intracranial aneurysm. As the physical functions of elderly patients are in a degraded state, their tolerance to injury and repair function are poor, which results in an increase in the incidence of adverse events. According to prior research, hypertension is one risk factor of intracranial aneurysmal SAH [25]. Huang et al. [26] have also found that patients given antihypertensive drugs face a lower risk of aneurysm formation. The results suggest the necessity to pay attention to controlling blood pressure and giving health education for patients, which are helpful in improving the prognosis of patients.

Our study has confirmed through analysis that TTM + motivational interviewing has a positive effect on improving self-management behaviour and QoL of patients with intracranial aneurysm. However, the present study still has some limitations. In such a retrospective study, the analysis of data results is probably biased. Secondly, due to the limited time, the adverse events of patients within only 6 months were tracked through outpatient reexamination and electronic medical records, and the long-term adverse events of patients were still not clear. Therefore, we hope to carry out more research and collect more samples in the follow-up research to supplement our research conclusions.

## 5. Conclusion

To sum up, TTM + motivational interviewing can help improve the self-management behaviour and QoL of patients with intracranial aneurysm without increasing the occurrence of adverse events, so it is worthy of clinical application.

## Figures and Tables

**Figure 1:** Changes of self-management behaviour scores in patients prior- and post-therapy. (a) Changes of symptom management scores of the two groups prior- and post-therapy. (b) Changes of daily life management scores of the two groups prior- and post-therapy. (c) Changes of emotional management scores of the two groups prior- and post-therapy. (d) Changes of social management scores of the two groups prior- and post-therapy. (e) Changes of data utilization management scores of the two groups prior- and post-therapy. (f) Changes of diet management scores of the two groups prior- and post-therapy. Note. Independent sample *t*-test was adopted for intergroup comparison, and paired *t*-test for intro-group comparison, ^*∗∗*^*P* < 0.01, ^*∗∗∗*^*P* < 0.001.

RETRACTED

**Figure 2:** Changes of SF-36 scores of patients prior and post-therapy. (a) Changes of mental health scores of the two groups prior- and post-therapy. (b) Changes of physiological health scores of the two groups prior- and post-therapy. (c) Changes of physical activity scores of the two groups prior- and post-therapy. (d) Changes of emotional function scores of the two groups prior and post-therapy. (e) Changes of social relations scores of the two groups prior- and post-therapy. (f) Changes of vitality scores of patients in the two groups prior- and post-therapy. Note: Independent sample *t*-test was adopted for intergroup comparison, and paired *t*-test for intro-group comparison, ^*∗∗*^*P* < 0.01, ^*∗∗∗*^*P* < 0.001.

**Figure 3:** ROC curves of age, history of hypertension, and combination of them in predicting adverse events. (a) ROC curve of age in predicting adverse events. (b) ROC curve of history of hypertension in predicting adverse events. (c) ROC curve of age + history of hypertension in predicting adverse events.

**Table 1:** Contents of motivational interviewing in each stage.

Stage	Target	Time	Mode	Content
Preintention stage (7 days after admission)	Establish willingness	40–60 min	Face-to-face interview in ward	The emphases were placed on mutual understanding, establishment of trust relationship, informing of research purpose, implementation of intervention, and informing of the correlation between bad behaviours and diseases.
Intention stage (8–14 days after admission)	Give support	20–30 min	Face-to-face interview in ward	The emphases were placed on the ways to promote healthy behaviour change and enhance confidence in it to discuss the difficulties and solutions in the process of behaviour change.
Preparation stage (3 days before discharge)	Promote confidence	20–30 min	Face-to-face interview in ward	The emphases were placed on jointly analyzing the life changes and benefits of healthy diet and regular exercise for patients, improving patients' confidence and determination to adhere to healthy behaviours, and maintaining healthy behaviours. Efforts were made to understand the patients' behaviour, and the patients were encouraged to sign the behaviour change agreement and were guided in making daily recording based on the Health Care Book for Patients with Intracranial Aneurysm (self-made).
Action stage (within 1 month after discharge)	Cultivate habits	20–30 min	Follow-up by telephone	Efforts were made to understand the habit maintenance and existing problems of patients' behaviour stage and give targeted guidance and consolidation. The patients were instructed to keep records based on the Health Book for Patients with Intracranial Aneurysm.
Maintenance stage (2-3 months after discharge)	Maintain habits	20–30 min	Follow-up by telephone	Efforts were made to understand the maintenance situation and existing problems of patients' behaviour stage, observe habit maintenance, and give targeted guidance and consolidation. The patients were instructed to keep records based on the Health Book for Patients with Intracranial Aneurysm.

RETRACTED

**Table 2:** Baseline data of patients (*n*(%)).

Index	The control group (*n* = 45)	The observation group (*n* = 49)	*χ* ^2^	*P* value
Age (years)			0.096	0.756
≥45	28 (62.22)	32 (65.31)		
<45	17 (37.78)	17 (34.69)		

Gender			0.310	0.577
Male	25 (55.56)	30 (61.22)		
Female	20 (44.44)	19 (38.78)		

BMI (kg/m^2^)			0.745	0.106
≥22	27 (60.00)	31 (63.27)		
<22	18 (40.00)	18 (36.73)		

Past medical history				
History of hypertension	12 (26.67%)	15 (30.61)	0.178	0.673
Diabetes mellitus	8 (17.78)	10 (20.41)	0.105	0.764

Location of intracranial aneurysm			0.652	0.722
Anterior circulation	26 (57.78)	32 (65.30)		
Posterior circulation	11 (24.44)	9 (18.37)		
Anterior and posterior circulation	8 (17.78)	8 (16.33)		

Note. Chi-square test was adopted for data analysis. BMI, body mass index.

**Table 3:** Comparison of BI and MOCA scores of patients prior- and post-treatment.

Groups	BI		*t*	*P* value	MOCA score		*t*	*P* value
	Before treatment	After treatment			Before treatment	After treatment		
The observation group (*n* = 49)	43.10 ± 7.81	93.02 ± 4.30	33.950	<0.001	23.14 ± 2.39	26.91 ± 2.01	7.731	<0.001
The control group (*n* = 45)	41.57 ± 8.9	81.28 ± 7.42	25.882	<0.001	23.44 ± 2.92	24.93 ± 2.07	2.976	0.020
*t* value	1.014	7.807			0.604	4.053		
*P* value	>0.05	<0.001			>0.05	0.004		

Note. Independent sample *t*-test was adopted for intergroup comparison, and paired *t*-test for intro-group comparison.

**Table 4:** Comparison of adverse events.

Groups	Intracranial hemorrhage	Progressive ischemic stroke	Recurrence of aneurysm	Died	Total incidence rate
The observation group (*n* = 49)	1	2	1	1	5 (10.20%)
The control group (*n* = 45)	3	3	3	2	11 (24.44%)
*χ* ^2^ value	1.232	0.311	1.232	0.439	3.368
*P* value	0.267	0.577	0.267	0.508	0.067

Note. Chi-square test was adopted for data analysis.

RETRACTED

**Table 5:** Assignment.

Factor	Assignment
Age (*X*)	≥45 = 1, <45 = 0
Gender (*X*)	Male = 1, female = 0
BMI (*X*)	≥22 kg/m^2^ = 1, <22 kg/m^2^ = 0
History of hypertension (*X*)	Yes = 1, No = 0
Diabetes mellitus (*X*)	Yes = 1, No = 0
Location of intracranial aneurysm (*X*)	The anterior circulation = 0, the posterior circulation = 1, and the anterior and posterior circulation = 2.
Intervention plan (*X*)	TTM + Motivational interviewing = 0, traditional management = 1
Incidence of adverse events (*Y*)	Yes = 0, No = 1

Note. *X*, Independent variable; *Y*, Dependent variable.

**Table 6:** Logistics regression analysis.

Factor	Univariate analysis			Multivariate analysis		
	*P* value	OR value	95% CI	*P* value	OR value	95% CI
Age	0.023	11.00	1.383–87.477	0.014	15.806	1.507–123.161
Gender	0.020	0.255	0.080–0.807	0.174	0.384	0.097–1.525
BMI	0.623	0.761	0.256–2.262			
History of hypertension	<0.001	12.600	3.560–44.596	<0.001	16.199	4.114–63.784
Diabetes mellitus	0.185	2.273	0.675–7.647			
Location of intracranial aneurysm	0.444	1.298	0.666–2.532			
Therapeutic regimen	0.074	2.847	0.903–8.973			

**Table 7:** ROC parameter.

Parameter	AUC	95 CI%	*P* Value	Specificity (%)	Sensitivity (%)
Age	0.680	0.557∼0.804	0.024	93.75	42.31
History of hypertension	0.779	0.645∼0.912	0.001	75.00	80.77
Unite	0.851	0.751∼0.952	<0.001	59.78	91.03

Note. AUC, area under curve.

## Data Availability

The labeled dataset used to support the findings of this study are available from the corresponding author upon request.

## References

[1] Sharma D. (2020). Perioperative management of aneurysmal subarachnoid hemorrhage. *Anesthesiology*.

[2] Yokosuka J., Fukaya S., Yamomoto S., Ueki K., Kim P. (2020). Intracranial subarachnoid hemorrhage caused by an aneurysm at the thoracic spinal region: case report and literature review. *British Journal of Neurosurgery*.

[3] Gathier C. S., van den Bergh W. M., van der Jagt M. (2018). Induced hypertension for delayed cerebral ischemia after aneurysmal subarachnoid hemorrhage: a randomized clinical trial. *Stroke*.

[4] Hashemzadeh M., Rahimi A., Zare-Farashbandi F., Alavi-Naeini A. M., Daei A. (2019). Transtheoretical model of health behavioral change: a systematic review. *Iranian Journal of Nursing and Midwifery Research*.

[5] Tseng H. M., Liao S. F., Wen Y. P., Chuang Y. J. (2017). Stages of change concept of the transtheoretical model for healthy eating links health literacy and diabetes knowledge to glycemic control in people with type 2 diabetes. *Primary Care Diabetes*.

RETRACTED

[6] Shinitzky H. E., Kub J. (2001). The art of motivating behavior change: the use of motivational interviewing to promote health. *Public Health Nursing*.

[7] Bassilios B., Judd F., Pattison P., Nicholas A., Moeller-Saxone K. (2015). Predictors of exercise in individuals with schizophrenia: a test of the transtheoretical model of behavior change. *Clinical Schizophrenia and Related Psychoses*.

[8] Li X., Yang S., Wang Y., Yang B., Zhang J. (2020). Effects of a transtheoretical model - based intervention and motivational interviewing on the management of depression in hospitalized patients with coronary heart disease: a randomized controlled trial. *BMC Public Health*.

[9] Thompson B. G., Brown R. D., Amin-Hanjani S. (2015). American heart association stroke council CoC, stroke N, council on E, prevention, American heart A and American stroke A. Guidelines for the management of patients with unruptured intracranial aneurysms: a guideline for healthcare professionals from the American heart association/American stroke association. *Stroke*.

[10] Lins L., Carvalho F. M. (2016). SF-36 total score as a single measure of health-related quality of life: scoping review. *SAGE Open Medicine*.

[11] Prodinger B., Oâ€™Connor R., Stucki G., Tennant A. (2017). Establishing score equivalence of the functional independence measure motor scale and the Barthel index, utilising the international classification of functioning, disability and health and rasch measurement theory. *Journal of Rehabilitation Medicine*.

[12] Carson N., Leach L., Murphy K. J. (2018). A re-examination of montreal cognitive assessment (MoCA) cutoff scores. *International Journal of Geriatric Psychiatry*.

[13] Thompson J. W., Elwardany O., McCarthy D. J. (2019). In vivo cerebral aneurysm models. *Neurosurgical Focus*.

[14] Jiang B., Paff M., Colby G. P., Coon A. L., Lin L. M. (2016). Cerebral aneurysm treatment: modern neurovascular techniques. *Stroke and Vascular Neurology*.

[15] Starke R. M., Chalouhi N., Ali M. S. (2013). The role of oxidative stress in cerebral aneurysm formation and rupture. *Current Neurovascular Research*.

[16] Czekajlo A. (2019). Role of diet-related factors in cerebral aneurysm formation and rupture. *Roczniki Panstwowego Zakladu Higieny*.

[17] Kwon O. K. (2019). Headache and aneurysm. *Neuroimaging Clinics of North America*.

[18] Scott L., Andrewes T. (2021). Using the transtheoretical model of behaviour change to analyse the impact of stopping exercise: a reflection. *British Journal of Nursing*.

[19] Watakakosol R., Suttiwan P., Ngamake S. T. (2021). Integration of the theory of planned behavior and transtheoretical model of change for prediction of intentions to reduce or stop alcohol use among Thai adolescents. *Substance Use & Misuse*.

RETRACTED

[20] de Freitas P. P., de Menezes M. C., Dos Santos L. C., Pimenta A. M., Ferreira A. V. M., Lopes A. C. S. (2020). The transtheoretical model is an effective weight management intervention: a randomized controlled trial. *BMC Public Health*.

[21] Ream E., Gargaro G., Barsevick A., Richardson A. J. P. E., Counseling (2015). Management of cancer-related fatigue during chemotherapy through telephone motivational interviewing: modeling and randomized exploratory trial. *Patient Education and Counseling*.

[22] Shirazi K. K., Wallace L. M., Niknami S. (2007). A home-based, transtheoretical change model designed strength training intervention to increase exercise to prevent osteoporosis in iranian women aged 40–65 years: a randomized controlled trial. *Health Education Research*.

[23] Rubak S., Sandbaek A., Lauritzen T., Christensen B. (2005). Motivational interviewing: a systematic review and meta-analysis. *The British Journal of General Practice*.

[24] Fahey K. F., Rao S. M., Douglas M. K., Thomas M. L., Elliott J. E., Miaskowski C. (2008). Nurse coaching to explore and modify patient attitudinal barriers interfering with effective cancer pain management. *Oncology Nursing Forum*.

[25] Marcolini E., Stretz C., DeWitt K. M. (2019). Intracranial hemorrhage and intracranial hypertension. *Emergency Medicine Clinics of North America*.

[26] Huang C., Li Z. Q. (2016). Factors affecting the prognosis of ruptured intracranial aneurysm. *Chinese Journal of Geriatrics|Chin J Geriatr*.

